# Antibiotic-Resistant Bacteria and Resistance Genes in Isolates from Ghanaian Drinking Water Sources

**DOI:** 10.1155/2022/2850165

**Published:** 2022-10-06

**Authors:** Stephen T. Odonkor, Shirley Victoria Simpson, William R. Morales Medina, N. L. Fahrenfeld

**Affiliations:** ^1^School of Public Services and Governance, Ghana Institute of Management and Public Administration, Accra, Ghana; ^2^Noguchi Memorial Institute for Medical Research LG 581, Legon-Accra, Ghana; ^3^Microbiology & Molecular Genetics, Rutgers, The State University of New Jersey, Piscataway, NJ, USA; ^4^Civil & Environmental Engineering, Rutgers, The State University of New Jersey, Piscataway, NJ, USA

## Abstract

The control of infectious diseases is seriously threatened by the increase in the number of microorganisms resistant to antimicrobial agents. Antibiotic-resistant bacteria have also been identified in the water environment. A field study was performed sampling drinking water sources in seven districts of southern Ghana targeting boreholes, dams, hand-dug wells, and streams during baseflow conditions. Bacteria were isolated (*N* = 110) from a total of 67 water samples to investigate their antimicrobial susceptibility and to determine their carriage of select antibiotic resistance genes. Bacterial identification was performed using conventional selective media methods and the analytical profile index (API) method. Antibiotic susceptibility tests were carried out using the Kirby–Bauer method. Results indicated that all water sources tested were of poor quality based on the presence of fecal indicator organisms. The most commonly occurring bacterium isolated from water was *Klebsiella* spp. (*N* = 24, 21.8%), followed by *E. coli* (*N* = 23, 20.9%). Gram-negative bacteria isolates were most commonly resistant to cefuroxime (24.5%), while the Gram-positives were most commonly resistant to meropenem (21.3%). The highest rates of bacterial resistances to more than one antibiotic were observed in *Klebsiella* spp. (30.0%) followed by *E. coli* (27.8%). PCR was used to detect the presence of a select antibiotic resistance genes in the Gram-negative isolates. The presence of *bla*_NDM-1_, *sul*l, *tet*(O), and *tet*(W) were observed in isolates from all water sources. In contrast, *erm*F was not detected in any of the Gram-negative isolates from any water source. Most (28.7%) of the resistance genes were observed in *E. coli* isolates. Reducing microbial contamination of the various water sources is needed to protect public health and to ensure the sustainability of this resource. This further calls for education of the citizenry.

## 1. Introduction

Good quality water is vital for human health, which directly relates to the socioeconomic progress of a country [8, 78]. It is also critical towards the attainment of UN Sustainable Development Goal (SDG) number six, which is aimed at ensuring the availability and sustainable management of water and sanitation for all. However, clean fresh water today is a scarce resource, particularly in the developing world. Globally, 663 million people do not have access to safe water [23]. Rural communities in Sub-Saharan Africa account for more than 50% of those people [27, 57]. Most of these communities, therefore, rely on untreated sources such as streams, dams, boreholes, wells, and rivers to meet fundamental needs such as drinking, sanitation, cooking, and for their sustainable development [54, 58]. Ghana missed the United Nations Millennium Development target on sanitation [11], which has a direct impact on food safety and security as well [40].

The global burden of waterborne disease is further complicated by climate change altering the patterns of disease, and more importantly by the increasing occurrences of antibiotic resistance observed both in the clinic and in the water environment (Gimelli, et al., 2018). Antibiotic-resistant genes (ARGs) conferring resistance to a wide variety of antibiotics have been identified in a large range of water environments, including drinking water in both developed and developing countries (e.g., [42, 46]. The major risk for public health is that resistance genes can be transferred from environmental bacteria to human pathogens. With this, antimicrobial resistance has become an important public health issue globally [14, 64]. Antimicrobial-resistant bacteria (ARB) and ARGs have therefore been considered environmental contaminants with widespread distribution in various environments, including water sources and drinking water systems [14, 77]. Importantly, the rapid and widespread increase of new ARB and ARGs all over the world has accelerated in recent years often associated with an increase in the discharge of antibiotics and other pollutants into the environment [64]; Schafhauser et al., 2015). In light of this, antimicrobial resistance has become an important theme in environmental and health science.

Several studies in Sub-Saharan African countries have reported the presence of antibiotic-resistant strains of bacteria, all showing high levels of resistance to antimicrobial agents [25, 39, 72]. In Ghana specifically, there is some evidence of increasing bacteria resistance to antibiotics. However, these data are skewed towards clinical isolates [28, 48, 79]. Thus, there is a paucity of data on environmental antibiotic resistance. It is worth noting that in Ghana, antibiotics are readily available over the counter without a doctor's prescription. Antibiotics are widely used in agriculture, particular for livestock rearing [79].

Unfortunately, environmental monitoring in Ghana is hardly part of the treatment and advocacy process for these diseases, nor for water quality. This surveillance is critical to public health and safety, as it contributes and supports improvements in water quality and antimicrobial resistance control (Hope et al., 2020; Gara, et al., 2018.) Furthermore, antimicrobial resistance (AMR) data could inform decisions and raise awareness among stakeholders and policymakers. Surveillance of AMR under a ‘One Health' framework is thus needed to provide data for awareness and decision making and to enhance understanding of links between environmental and clinical AMR. Therefore, the objectives of this study were as follows: (1) determine the occurrence and identity of bacteria in Ghanaian drinking water sources, (2) determine antibiotic susceptibility profiles of the bacterial isolates, and (3) determine the resistance genes associated with the bacteria.

## 2. Material and Methods

### 2.1. Sample Collection Sites

Seven communities were then identified and selected for sampling after several preliminary visits were made to communities across the study area (Figure 1). The sampling sites in each community comprised of four different water sources as follows: boreholes (typical depths > 5 m to 50m), dams, hand-dug wells (typical depths < 1 m to 3 m), and streams.  Table 1 shows details of the water sampled.

Sample sites were chosen to be representative of community water sources based primarily on factors such as popular water locations, extent of usage, and level of patronage of water from these sources. Prior to water sampling, observations were made around the sampling sites. These observations included the sanitary conditions, as well as possible sources of contamination which could influence water quality from the sources sampled. Field records for environmental factors, presence of animals, and fecal accidents, among others, were noted.

### 2.2. Sample Size and Sampling Frequency

A total of sixty-seven composite water samples were collected for assessment. One liter of water was collected in each sample. Water samples were taken in duplicates from each sample site to form the composite sample for analysis. All water sampling and preservation procedures were performed according to Standard Methods for the Examination of Water and Wastewater [9, 10] and WHO guidelines for drinking water quality [16, 33]. Sampling for bacteriological analysis was performed aseptically. Field blanks consisted of autoclaved distilled water, carried into the field, and analyzed to ensure that the samples were not contaminated during the sampling process. All samples were transported on ice to the laboratory within 2 hours.

### 2.3. Bacterial Isolation and Identification

Isolates from overnight cultures of the water samples were further characterized by streaking on MacConkey agar and incubated overnight at 37°C. This was done to obtain pure isolates prior to identification. All Gram-positive bacteria were identified by conventional methods including Gram stain, positive catalase, tube coagulase, and deoxyribonucleases (DNAse) test [32]. An API 20E kit was used to identify and differentiate the Gram-negative bacteria of the family Enterobacteriaceae following the manufacturer's instructions.

### 2.4. Antibacterial Susceptibility Testing

Each of the bacterial isolates was subjected to antibiotic susceptibility testing using the Kirby–Bauer method that has been standardized and evaluated by the methods of Clinical and Laboratory Standards Institute (CLSI) [30]. Isolates grown overnight on nutrient agar were suspended in sterile normal saline (0.9% *w*/*v* NaCl) using a sterile wire loop until the turbidity was equal to 0.5 Mcfarland standards. Sterile nontoxic cotton swabs dipped into the standardized inoculum were used to streak the entire surface of Mueller–Hinton agar plates. Gram-positive bacteria were tested against 12 antibiotics as follows: ampicillin (10 *μ*g), cloxacillin (10 *μ*g), erythromycin (15 *μ*g), tetracycline (30 *μ*g), cotrimoxazole (25 *μ*g), cefuroxime (30 *μ*g), gentamicin (10 *μ*g), penicillin (10 IU), ciprofloxacin (5 *μ*g), augmentin (30 *μ*g), vancomycin (30 *μ*g), and meropenem (25 *μ*g). Gram-negative bacteria were tested against 11 antibiotics as follows: ampicillin (10 *μ*g), tetracycline (30 *μ*g), cotrimoxazole (25 *μ*g), cefuroxime (30 *μ*g), chloramphenicol (30 *μ*g), ceftriaxone (25 *μ*g), cefotaxime (30 *μ*g), ciprofloxacin (5 *μ*g), amikacin (30 *μ*g), vancomycin (30 *μ*g), and meropenem (25 *μ*g). Antibiotic disks were aseptically placed using sterile forceps, and all plates were incubated at 37°C for 24 hrs. The results were interpreted using CLSI [76]. The susceptibility testing was repeated for each isolate to ensure that the results obtained were consistent.

### 2.5. DNA Extraction and PCR

Bacterial cultures stored Mueller–Hinton broth were extracted for identification of ARGs. To extract DNA, 1 mL of the suspension was transferred into a test tube containing 1 mL of sterile molecular biology grade deionized water (ddH_2_O) and heat shocked for 10 minutes at 95°C in a water bath. A negative control of ddH_2_O was simultaneously processed and tested to assess possible contamination during the DNA extraction. The solution was then centrifuged for five minutes at 14,000 × g. The supernatant containing bacterial DNA was transferred to a new 2 mL tube and stored at -20°C for downstream molecular analysis.

Polymerase chain reaction (PCR) targeting the bacterial 16S rRNA gene (Table 2) was used to confirm the DNA extraction method. PCR targeting eight different ARGs (*erm*F, *mex*B, bla*_ndm1_*, *sul*1, *sul*2, *tet*(G), *tet*(O), and *tet*(W)) was used to determine the presence or absence of each gene in all Gram-negative bacterial isolates. *ermF* encodes for macrolide resistance, *mex*B for a multidrug efflux pump, bla*_ndm1_* encodes for a metallobetalactamase, the *sul* genes for sulfonamide resistance, and the *tet* genes for resistance to tetracycline antibiotics. These genes were chosen to represent a range of resistance types including some that are commonly observed (i.e., *sul* and *tet* genes) in environmental matrices and some of high medical relevance (i.e., bla*_ndm1_*). The PCR mixture for each reaction contained 12.5 *μ*L of 2 × Taq PCR Master Mix ((0.1 U Taq polymerase/*μ*L, 0.5 mM dNTP, and 3 MgCl_2_,), 0.5 *μ*L of each primer (1 *μ*M), 1 *μ*L of template DNA, and ddH_2_O to a final volume of 25 *μ*L. No template controls were performed during each PCR reaction. Positive controls were comprised of 1 *μ*L containing 10^5^ copies of DNA standards for each ARG, quantified with gel electrophoresis. PCR thermocycler condition and primer sequences for each ARG and the 16S rRNA gene are summarized in Table 2. The presence or absence of a given target gene was assessed through observation of the expected amplicon length (determined using a DNA ladder) via gel electrophoresis.

### 2.6. Statistical Analysis

All the statistical analyzes were performed in R (R Team, 2018). To compare the genomic antibiotic resistance profile as a factor water sources, a value of one was assigned to the detected genes and a value of zero was assigned to the nondetected genes to create a presence/absence antibiotic resistance profile for each isolate. Statistical differences were determined through a permutational multivariate analysis of variance (PERMANOVA) and a *post hoc* pairwise PERMANOVA with a Bonferroni *p* adjustment: Pairwise Adonis package version 0.3 [12, 34]. Differences in multiple antibiotic resistance (MAR) indices as a factor of water source were evaluated using a Kruskal–Wallis test with a *post hoc* pairwise *t*-test with a Bonferroni correction for multiple comparisons. Nonnormality of the data was confirmed by a Shapiro-Wilk test.

## 3. Results

A total of 110 bacteria isolates were obtained across all of the water sources sampled during the period of study (Table 3). The most commonly occurring bacterium isolated from the water samples was *Klebsiella* spp. with 24 isolates (21.8% of total study isolates). The second most commonly observed bacteria was *E. coli.* with 23 isolates (20.9% of total study isolates). The highest number of bacterial isolates were obtained from stream water sources with 42 isolates obtained (38.2% of total study isolates), while the least were isolated from borehole water sources with nine isolates (8.2% of the total study isolates).

The antibiotic resistance profiles observed are presented in Tables 4 and 5 for Gram-negative and Gram-positive bacteria isolated, respectively. Similar MAR values were detected among the isolated bacterial taxa with *N* = 3 or higher (*p* > 0.14, pairwise *t*-test) The Gram-negative bacterial isolates were most commonly resistant to CRX (cefuroxime) (24.5%) followed by cefotaxime and MEM (meropenem) with each exhibiting 21.3% resistance. *Klebsiella* spp. isolates had phenotypic resistance most often (30.0%) followed by *Escherichia coli* (27.8%). The Gram-positive bacterial isolates were commonly resistant to MEM (21.3%) followed by VAN and AUG (both 17%). Among these isolates, multidrug resistance was most common among *S. aureus* (59.6%) and *S. epidermis* (36.2%).

MAR indices of the bacterial isolates were determined for the various water sources (Table 6). The multiple antibiotic resistance (MAR) index is defined as *a*/*b*, where *a* represents the number of antibiotics to which the isolate was resistant and *b* represents the number of antibiotics to which the isolate was subjected. The aggregate MAR index for a sampling sources (MAR *q*) is defined as the ratio between the number of resistant tests at the sampling sources and the total number of tests performed at the sampling source. Stream water sources recorded the highest MAR *q* values of 0.9. This was followed by a MAR *q* for the dam water sources which was 0.8 and hand-dug well water sources with a recorded value of 0.6. Stream water sources resulted in a significantly higher MAR value than hand-dug well (*p* = 0.01, pairwise *t*-test); however, no other differences were detected as in MAR values as a factor of source.

The presence of eight (8) different antibiotic resistance genes were tested for each Gram-negative bacterium isolated from the samples using PCR amplification (Table 7). *bla*_NDM-1_, *sul*1, *tet*(O), and *tet*(W) resistance genes were detected in isolates collected from all water sources, while *erm*F was not detected in isolates from any of the water sources. The number of genes amplified from isolates from each water source is presented in Table 7. All water sources resulted in a similar antibiotic resistance profile (*p* = 1; pairwise PERMANOVA) except for dam compared to the hand-dug well which resulted in a significantly different profile (*p* < 0.006; pairwise PERMANOVA). The MAR index was similar among all water sources (*p* > 0.16; pairwise *t*-test).

An inventory of ARGs identified in the bacterial isolates is presented in Table 8. Note that most (28.7%) of the resistance genes were obtained from *Escherichia coli (E. coli)* isolates. This was followed by *Klebsiella* spp. with 27.6%. *Enterobacter* spp. accounted for 12.6% of the resistance genes observed, representing the third highest. The most frequently detected ARG was *sul*1, which was observed in 46% of isolates tested. This was followed by *bla*_NDM-1_, identified in 35.1% of isolates tested.

## 4. Discussion

### 4.1. Isolate Observations and Implications for Microbial Water Quality

In the present study, several bacteria of public health importance were identified in Ghanaian water sources: *Salmonella* spp. (typhoid fever and acute diarrheal infection), *Vibrio* spp. (cholera), and *Klebsiella* spp. (pneumonia and urinary/lower biliary tract disease [62]). *Vibrio* spp. and *Klebiella* spp. were isolated from each water source type in the present study while *Salmonella* spp. were isolated from the streams. Similar reports of the isolation of these organisms were made by Moges et al. [47] and also by Shahina et al. [69], from an assessment of ground and surface water sources in India.

The most commonly isolated bacteria were *E. coli* which were isolated from each type of water source. While the aim of this study was not quantifying *E. coli* in the water sources, it is worth noting that detection of one *E. coli* CFU per 100 mL is in exceedance of the World Health Organization's guidance values for water intended for drinking [73]. *E. coli* is widespread in the environment but elevated levels are indicative of fecal pollution [29] and the prevalence of water-related gastroenteritis [61]. While most *E. coli* strains are not pathogenic, given that some strains are pathogenic they have been used for disease risk assessment [53]. Recent studies have shown that rural water sources in Ghana have high occurrences of coliforms [49, 51, 55], another fecal indicating organism. Similarly, Nogueira et al. *[*50*]* reported that untreated water sources were more deeply contaminated with fecal coliforms than treated water sources.

### 4.2. Antimicrobial Resistance among Isolates

The current study also evaluated both phenotypic and genotypic antibiotic resistance among the waterborne isolates. Phenotypically, we observed multiple antibiotic resistance in both Gram-positive and Gram-negative isolates to commonly used antibiotics in the study area [4, 38]. These antibiotics include ampicillin, cloxacillin, erythromycin, tetracycline, cotrimoxazole, cefuroxime, gentamicin, penicillin, ciprofloxacin, augmentin, vancomycin, meropenem, chloramphenicol, ceftriaxone, amikacin, and meropenem [38]. Data from hospital surveys [38] in rural Ghana indicate that two of the antibiotics tested here were among top five most frequently prescribed (i.e., ceftriaxone and cefuroxime). Despite legal COT sales over-the-counter in Ghana, COT resistance was observed at a lower prevalence than several other antibiotics tested. The fact that illegal sales of other antibiotics from Licensed Chemical Sellers is known [4] may explain why the most available antibiotic was not associated with the most commonly observed phenotypic resistance.

In terms of Gram-positive isolates, *S. aureus* accounted for 59.6% of all multidrug resistances observed in the Gram-positive isolates. *S. aureus* also had a high MAR value of 2.3. *S. aureus* isolates were resistant to 12 of the antibiotics it was tested against, all except gentamicin. Multidrug-resistant *S. aureus* occurs commonly and has been observed in several diverse environments, including drinking water and food, indicating an important public health concern [2].

Multiple drug resistance was also commonly observed in Gram-negative bacteria. *Klebsiella* spp. and *Escherichia coli* showed a high prevalence of resistance to cefuroxime and cefotaxime. Likewise, a high prevalence of resistance to cefuroxime and cefotaxime has been recorded from clinical isolates in Ghana [5, 37]: [56]. We observed low resistance to ampicillin in contrast to findings from Moges et al. [47] who observed all isolates of *Klebsiella* spp. and *Escherichia coli* were resistant to ampicillin. Interestingly, we did not observe any bacterial resistance to ciprofloxacin. This observation is in contrast to another study done in Bangladesh, where 100% of waterborne Gram-negative bacteria isolates were resistant to ciprofloxacin [31], and in a similar study in Nigeria, where 54.7% of Gram-negative isolates obtained from water were found to resistant to ciprofloxacin (Ojayi and Ojo 2018).

In this current study, we also investigated the aggregate MAR index for sampling sources (MAR *q*). A number of factors could be responsible for the resistance observed at the sampling sites. For example, we made an interesting observation of the presences of two bacteria of public health importance *Shigella* spp. and *Salmonella typhi*, known to cause dysentery and typhoid fever/acute diarrheal infection, respectively [63] from ground water sources (boreholes and hand-dug wells). After a careful assessment of location, we discovered that the boreholes and hand-dug wells in question were likely contaminated with these enteric bacteria from the rural public ground toilet systems that were situated at an average of 50 meters from the location of those ground water sources sampled.

The MAR indices of isolates from surface water sources were comparable with those of previous studies [7, 17, 60]. Similar to the results presented here, Tambekar et al. [70] reported high MAR indices due to human and nonhuman fecal contamination of surface, ground, and public supply water sites in Akola and Buldhana of Vidarbha district. Likewise, a similar study by Chatterjee et al. [19] noted that drinking water sources of Uttarakhand region were contaminated with high MAR index *E. coli* originating from potential risk sources.

### 4.3. Antimicrobial Resistance among Isolates

PCR was performed to detect the presence of eight ARGs. The genes were determined for each Gram-negative bacterium isolated and for each sampled water source (Table 6). *sul*1 and *bla_NDM-1_* resistance genes was found to be prevalent in isolates (46% and 31%, respectively) from all sampled water sources. The high prevalence of *sul*1 is not surprising; this gene is frequently observed in bulk environmental samples thus a suggested target for monitoring efforts (Vikesland et al., 2017). Tetracycline-resistant genes *tet*(O) and *tet*(W) were infrequently observed in isolates across water sources, which is contrast with similar studies by Chee-Sanford et al. [20] where *tet*(O) and *tet*(Q) were found to be regularly present in resistance isolates from water sources. However, in another study by Adesoji et al. [3], *tet*(O) was not detected in any of the isolates from water sources. Of particular interest is the frequent observation of the *bla*_NDM-1_ gene (35.1% of tested isolates). The *bla*_NDM-1_ gene is known to be transferred between bacterial genera ([36, 80] and has been reported in sewage and surface water isolates [36].

## 5. Conclusions

Bacteria associated with fecal contamination were observed in various water sources in the study communities. The study demonstrated multiple drug resistance to the commonly used antibiotics is high in rural communities in Ghana. Antibiotic-resistant bacteria were found to carry several antimicrobial-resistant genes. High MAR index values recorded in the study indicate a potential hazard associated with the sampled water sources, particularly the surface waters studied, potentially due poor sanitation contaminating the surface waters. This observation raises concern about water quality in rural Ghana and indicates a need to understand the sources of fecal and other contamination (i.e., human sewage) and opportunities for water treatment. Further investigation into the sources of the fecal microbes observed and measurements of resistance genes across in the source water microbiome could help provide further insight into the overall hazard posed by the waters tested and opportunities for mitigation. Future studies should include collection of other water quality parameters to understand any relationships between the water chemistry and ARGs or high MAR indices. Finally, the deployment of tools such as microbial source tracking for periodic monitoring of antibiotic sensitivity of the water sources is of importance to detect any changing patterns that may arise in the future. Further work in these areas may allow for the creation of more curative measures towards better management of water resources.

## Figures and Tables

**Figure 1:** Map of sampling communities and sampling location number (*L* number). Insert map shows location of the study area within Ghana.

**Table 1:** Composition of sampling locations and frequency.

Water source	Sampling locations							
	L1	L2	L3	L4	L5	L6	L7	Total
Borehole	2	2	2	2	2	2	2	14
Dam	2	2	2	2	2	3	3	16
Hand-dug well	3	2	2	3	2	3	3	18
Streams	2	2	3	3	3	3	3	19
Total	9	8	9	10	9	11	11	67

L1: Somanya; L2: Akuse; L3: Asutsuare; L4: New Ningo; L5: Old Ningo; L6: Odumase Krobo; L7: Dodowa.

**Table 2:** Primer sequences, PCR conditions, amplicon lengths for each ARG, and 16S rRNA gene.

Gene	Primer sequence (5′-3′)	PCR conditions	Amplicon length (bp)	Source
*sul*1	CGCACCGGAAACATCGCTGCAC	95°C for 2 m (98°C for 5 s, 69.9°C for 5 s) ×40 cycles	163	8
	TGAAGTTCCGCCGCAAGGCTCG			
*sul*2	TCC GGT GGA GGC CGG TAT CTG G	95°C for 2 m (98°C for 5 s, 65°C for 5 s) ×40 cycles	191	8
	CGG GAA TGC CAT CTG CCT TGA G			
*tet*(G)	GCAGAGCAGGTCGCTGG	98°C for 2 m (98°C for 5 s, 64°C for 5 s) ×40 cycles	134	9
	CCYGCAAGAGAAGCCAGAAG			
*erm*F	CGACACAGCTTTGGTTGAAC GGACCTACCTCATAGACAAG	95°C for 4 m (94°C for 30 s, 56°C for 30 s and 72°C for 30 s) ×40 cycles	309	10
*tet*(O)	ACGGARAGTTTATTGTATACC TGGCGTATCTATAATGTTGAC	98°C for 2 m (98°C for 5 s, 50°C for 5 s) ×40 cycles	171	12
*tet*(W)	GAGAGCCTGCTATATGCCAGC GGGCGTATCCACAATGTTAAC	98°C for 2 m (98°C for 5 s, 60°C for 5 s) ×40 cycles	168	12
bla_NDM-1_	TTTCAGTCCGACACAACGCG CAGCCACCAAAAGCGATGTC 6-FAM-CAACCGCGCCCAACTTTGGC-TAMRA	98°C for 15 m (98°C for 30 s, 59°C for 1 m) ×40 cycles	155	6
16S rRNA	CCTACGGGAGGCAGCAG ATTACCGCGGCTGCTGG	95°C for 10 m (95°C for 15 s, 60°C for 1 m) ×40 cycles	202	14

**Table 3:** Occurrence and distribution of bacteria isolated from the drinking water sources.

Bacteria	Boreholes	Dams	Hand-dug wells	Streams	Total	
					No.	(%)
*Acinetobacter* spp.	0	2	1	3	6	5.5
*Bacillus* spp.	0	0	1	0	1	0.9
*Citrobacter freundii*	0	1	0	1	2	1.8
*Enterobacter* spp.	1	3	2	5	11	10.0
*Enterococcus* spp.	0	1	0	0	1	0.9
*Escherichia coli*	3	7	4	9	23	20.9
*Klebsiella* spp.	1	9	2	12	24	21.8
*Proteus vulgaris*	0	1	0	1	2	1.8
*Providencia* spp.	0	1	0	1	2	1.8
*Pseudomonas aeruginosa*	0	2	**1**	2	5	4.5
*Salmonella* spp.	0	0	0	1	1	0.9
*Staphylococcus aureus*	3	4	5	4	16	14.5
*Staphylococcus epidermidis*	0	2	3	1	6	5.5
*Streptococcus agalactiae*	0	2	0	1	3	2.7
*Vibrio* spp.	1	2	3	1	7	6.4
Total	9 (8.2)^∗^	37 (33.6)	22 (20.0)	42 (38.2)	110	100.0

^∗^Number in parentheses represents the percent of the total isolates obtained.

**Table 4:** Antibiotic resistance patterns of Gram-negative bacteria isolated from the water sources.

Isolate	Pattern of antibiotic resistance: (number of resistant strains per antibiotic)											Multiple resistances		
	AMP	TET	COT	CRX	CHL	CTR	CTX	CIP	AMK	VAN	MEM	No.	%	MAR
*Acinetobacter* spp. (*n* = 6)	0	0	0	3	0	2	2	0	0	2	5	14	6.5	1.3
*Citrobacter freundii* (*n* = 2)	1	0	1	2	0	1	1	0	0	1	2	9	4.2	0.8
*Enterobacter* spp. (*n* = 11)	2	2	1	7	1	2	6	0	0	2	4	27	12.5	2.5
*Escherichia coli* (*n* = 23)	5	3	4	12	0	4	14	0	0	4	14	60	27.8	5.5
*Klebsiella* spp. (*n* = 24)	1	1	5	16	0	4	17	0	0	7	14	65	30.1	5.9
*Proteus vulgaris* (*n* = 2)	0	0	0	2	0	1	2	0	0	0	1	6	2.8	0.5
*Providencia* spp. (*n* = 2)	0	1	0	1	0	0	0	0	0	0	0	2	0.9	0.2
*Pseudomonas aeruginosa* (*n* = 5)	2	1	1	5	0	2	2	0	0	2	4	19	8.8	1.7
*Salmonella* spp. (*n* = 1)	0	1	0	1	0	1	1	0	0	1	1	6	2.8	0.5
*Vibro* spp. (*n* = 7)	1	0	1	4	0	0	1	0	0	0	1	8	3.7	0.7
Total	12 (5.6)	9 (4.2)	13 (6.0)	53 (24.5)	1 (0.5)	17 (7.9)	46 (21.3)	0 (0.0)	0 (0.0)	19 (8.8)	46 (21.3)	216	100	

Key: AMP: ampicillin; TET: tetracycline; CRX: cefuroxime; CHL: chloramphenicol; CTR: ceftriaxone; CTX: cefotaxime; CIP: ciprofloxacin; AMK: amikacin; VAN: vancomycin; MEM: meropenem.

**Table 5:** Antibiotic resistance patterns of Gram-positive bacteria isolated from the water sources.

Isolate	Pattern of antibiotic resistance: (number of resistant strains per antibiotic)												Multiple resistances		
	AMP	COX	ERY	TET	COT	CRX	GEN	PEN	CIP	AUG	VAN	MEM	No.	%	MAR
*Bacillus* spp. (*n* = 1)	0	0	0	0	0	0	0	0	0	0	0	0	0	0.0	0.0
*Enterococcus* spp. (*n* = 1)	0	0	0	0	0	0	0	0	0	0	0	0	0	0.0	0.0
*Staphylococcus aureus* (*n* = 16)	1	4	1	1	1	2	0	1	1	5	5	6	28	59.6	2.3
*Staphylococcus epidermidis* (*n* = 6)	0	3	0	1	0	3	0	0	0	3	3	4	17	36.2	1.4
*Streptococcus agalactiae* (*n* = 3)	0	0	0	0	0	2	0	0	0	0	0	0	2	4.3	0.2
Total	1 (2.1)	7 (14.9)	1 (2.1)	2 (4.3)	1 (2.1)	7 (14.9)	0 (0.0)	1 (2.1)	1 (2.1)	8 (17.0)	8 (17.0)	10 (21.3)	47	100	

Key: AMP: ampicillin; COX: cloxacillin; ERY: erythromycin; TET: tetracycline; COT: cotrimoxazole; CRX: cefuroxime; GEN: gentamicin; PEN: penicillin; CHL: chloramphenicol; CTR: ceftriaxone; CTX: cefotaxime; CIP: ciprofloxacin; AUG: augmentin; VAN: vancomycin; MEM: meropenem.

**Table 6:** Multiple antibiotic-resistant indexes of bacteria isolate at various water sources.

Water source	Total numbers of test (isolates)			No. of resistant test (resistant isolates)			MAR *q*
	Gram negative	Gram positive	Total	Gram negative	Gram positive	Total	
Borehole	6	3	9	5	1	6	0.7
Dam	29	8	37	26	3	29	0.8
Hand-dug well	13	9	22	12	2	14	0.6
Streams	36	6	42	31	5	36	0.9
Total	84	26	110	74	11	85	

MAR *q*: MAR index per sampling source.

**Table 7:** PCR detection of antibiotic resistance genes in DNA extracted from bacteria isolates at different water sources.

Water source	No. of test isolates	ARGs									
		*erm*F	*mex*B	*bla*_NDM-1_	*sul*1	*sul*2	*tet*(G)	*tet*(O)	*tet*(W)	Total	
										No.	%
Borehole	6	0	0	5	6	0	0	1	1	13	7.47
Dam	29	0	2	16	28	2	2	1	2	53	30.46
Hand-dug well	13	0	0	9	13	0	1	1	1	25	14.37
Streams	36	0	7	31	33	5	3	2	2	83	47.70
Total	84	0 (0.0)	9 (5.17)	61 (35.06)	80 (45.98)	7 (4.02)	6 (3.45)	5 (2.87)	6 (3.45)	174	100

**Table 8:** Inventory of antibiotic resistance genes identified in each bacteria isolate.

Isolate	ARGs								Total	
	*erm*F	*mex*B	*bla*_NDM-1_	*sul*1	*sul*2	*tet*(G)	*tet*(O)	*tet*(W)	No.	%
*Acinetobacter* spp.	0	0	5	6	0	0	1	0	12	6.9
*Citrobacter freundii*	0	1	1	2	0	1	0	0	5	2.9
*Enterobacter* spp.	0	1	9	11	0	1	0	0	22	12.6
*Enterococcus* spp.	0	0	0	1	0	0	0	0	1	0.6
*Escherichia coli*	0	3	17	23	2	1	1	3	50	28.7
*Klebsiella* spp.	0	2	17	22	1	3	2	1	48	27.6
*Proteus vulgaris*	0	1	0	2	0	0	0	0	3	1.7
*Providencia* spp.	0	0	2	2	0	0	0	0	4	2.3
*Pseudomonas aeruginosa*	0	1	4	5	0	0	1	1	12	6.9
*Salmonella* spp.	0	0	0	1	0	0	0	1	2	1.1
*Vibrio* spp.	0	0	6	5	4	0	0	0	15	8.6
Total	0	9	61	80	7	6	5	6	174	100.0

## Data Availability

The data used to support the findings of this study are included within the article.

## References

[1] Abdelgader S. A., Shi D., Chen M. (2018). Antibiotics Resistance Genes Screening and Comparative Genomics Analysis of Commensal _Escherichia coli_ Isolated from Poultry Farms between China and Sudan. *BioMed research international*.

[2] Abulreesh H. H. Multidrug-resistant staphylococci in the environment.

[3] Adesoji A. T., Ogunjobi A. A., Olatoye I. O., Douglas D. R. (2015). Prevalence of tetracycline resistance genes among multi-drug resistant bacteria from selected water distribution systems in southwestern Nigeria. *Annals of Clinical Microbiology and Antimicrobials*.

[4] Afari-Asiedu S., Kinsman J., Boamah-Kaali E. (2018). To sell or not to sell; the differences between regulatory and community demands regarding access to antibiotics in rural Ghana. *Journal of Pharmaceutical Policy and Practice*.

[5] Agyepong N., Govinden U., Owusu-Ofori A., Essack S. Y. (2018). Multidrug-resistant gram-negative bacterial infections in a teaching hospital in Ghana. *Antimicrobial Resistance & Infection Control*.

[6] Ojayi A. O., Ojo B. O. (2016). Antibiotics susceptibility profile of microorganisms encountered in riverine areas of Ondo state, Nigeria. *Journal of Disease and Global Health*.

[7] Akturk S., Dincer S., Toroglu S. (2012). Determination of microbial quality and plasmid mediated multidrug resistant bacteria in fountain drinking water sources in Turkey. *Journal of Environmental Biology*.

[8] Anthonj C., Diekkrüger B., Borgemeister C., Kistemann T. (2019). Health risk perceptions and local knowledge of water-related infectious disease exposure among Kenyan wetland communities. *International Journal of Hygiene and Environmental Health*.

[9] Apha (1995). *Standard Methods for the Examination of Water and Wastewater*.

[10] Apha (1998). *Standard Methods for the Examination of Water and Wastewater*.

[11] Appiah-Effah E., Duku G. A., Azangbego N. Y., Aggrey R. K. A., Gyapong-Korsah B., Nyarko K. B. (2019). Ghana's post-MDGs sanitation situation: an overview. *Journal of Water, Sanitation and Hygiene for Development*.

[12] Arbizu P. M. (2019). *pairwiseAdonis: pairwise multilevel comparison using adonis*.

[13] Bengtsson-Palme J., Larsson D. J. (2016). Concentrations of antibiotics predicted to select for resistant bacteria: proposed limits for environmental regulation. *Environment International*.

[14] Berendonk T. U., Manaia C. M., Merlin C. (2015). Tackling antibiotic resistance: the environmental framework. *Nature Reviews Microbiology*.

[15] Bergeron S., Raj B., Nathaniel R., Corbin A., LaFleur G. (2017). Presence of antibiotic resistance genes in raw source water of a drinking water treatment plant in a rural community of USA. *International Biodeterioration & Biodegradation*.

[16] Bürgmann H., Frigon D., Gaze W. H. (2018). Water and sanitation: an essential battlefront in the war on antimicrobial resistance. *FEMS microbiology ecology*.

[17] Chandran A., Hatha A. A. M., Varghese S., Sheeja K. M. (2008). Prevalence of multiple drug resistant Escherichia coli serotypes in a tropical estuary, India. *Microbes and Environments*.

[18] Chapman D. (1996). Water Quality Assessments. *A Guide to Use of Biota, Sediments and Water in Environmental Monitoring*.

[19] Chatterjee R., Sinha S., Aggarwal S. (2012). Studies on susceptibility and resistance patterns of various E. coli isolated from different water samples against clinically significant antibiotics. *Int. J Bioassays*.

[20] Chee-Sanford J. C., Aminov R. I., Krapac I. J., Garrigues-Jeanjean N., Mackie R. I. (2001). Occurrence and diversity of tetracycline resistance genes in lagoons and groundwater underlying two swine production facilities. *Applied and Environmental Microbiology*.

[21] Chen J., Li W., Zhang J. (2020). Prevalence of antibiotic resistance genes in drinking water and biofilms: the correlation with the microbial community and opportunistic pathogens. *Chemosphere*.

[22] Chitanand M. P., Kadam T. A., Gyananath G., Totewad N. D., Balhal D. K. (2010). Multiple antibiotic resistance indexing of coliforms to identify high risk contamination sites in aquatic environment. *Indian Journal of Microbiology*.

[23] Chitonge H., Mokoena A., Kongo M. (2020). Water and Sanitation Inequality in Africa: Challenges for SDG 6. *In Africa and the Sustainable Development Goals*.

[24] Das B. K., Behera B. K., Chakraborty H. J. (2020). Metagenomic study focusing on antibiotic resistance genes from the sediments of River Yamuna. *Gene*.

[25] Elton L., Thomason M. J., Tembo J. (2020). Antimicrobial resistance preparedness in sub-Saharan African countries. *Antimicrobial Resistance & Infection Control*.

[26] Ferrer N., Folch A., Masó G., Sanchez S., Sanchez-Vila X. (2020). What are the main factors influencing the presence of faecal bacteria pollution in groundwater systems in developing countries?. *Journal of Contaminant Hydrology*.

[27] Furtatova A., Kamenik L. (2018). Modeling features of sustainable urban development in modern conditions of water supply. *In MATEC Web of Conferences*.

[28] García-Vello P., González-Zorn B., Saba C. K. S. (2020). Antibiotic resistance patterns in human, animal, food and environmental isolates in Ghana: a review. *The Pan African Medical Journal*.

[29] Hachich E. M., Di Bari M., Christ A. P. G., Lamparelli C. C., Ramos S. S., Sato M. I. Z. (2012). Comparison of thermotolerant coliforms and Escherichia coli densities in freshwater bodies. *Brazilian Journal of Microbiology*.

[30] Hudzicki J. (2009). *Kirby-Bauer Disk Diffusion Susceptibility Test Protocol*.

[31] Islam M. J., Uddin M. S., Hakim M. A., Das K. K., Hasan M. N. (2008). Role of untreated liquid hospital waste to the development of antibiotic resistant bacteria. *J Innov Dev Strategy*.

[32] Ito T., Sekizuka T., Kishi N., Yamashita A., Kuroda M. (2019). Conventional culture methods with commercially available media unveil the presence of novel culturable bacteria. *Gut Microbes*.

[33] Jang J., Hur H. G., Sadowsky M. J., Byappanahalli M. N., Yan T., Ishii S. (2017). Environmental Escherichia coli: ecology and public health implications-a review. *Journal of Applied Microbiology*.

[34] Jari Oksanen F. G. B., Friendly M., Kindt R. (2019). Community ecology package. *R package version 2.5-6*.

[35] Krumperman P. H. (1983). Multiple antibiotic resistance indexing of Escherichia coli to identify high-risk sources of fecal contamination of foods. *Applied and Environmental Microbiology*.

[36] Kumarasamy K. K., Toleman M. A., Walsh T. R. (2010). Emergence of a new antibiotic resistance mechanism in India, Pakistan, and the UK: a molecular, biological, and epidemiological study. *The Lancet Infectious Diseases*.

[37] Labi A. K., Bjerrum S., Enweronu-Laryea C. C., Ayibor P. K., Nielsen K. L., Marvig R. L. (2020). *High carriage rates of multidrug-resistant gram-negative bacteria in neonatal intensive care units from Ghana*.

[38] Labi A. K., Obeng-Nkrumah N., Nartey E. T. (2018). Antibiotic use in a tertiary healthcare facility in Ghana: a point prevalence survey. *Antimicrobial Resistance & Infection Control*.

[39] Leopold S. J., van Leth F., Tarekegn H., Schultsz C. (2014). Antimicrobial drug resistance among clinically relevant bacterial isolates in sub-Saharan Africa: a systematic review. *Journal of Antimicrobial Chemotherapy*.

[40] Lu Y., Song S., Wang R. (2015). Impacts of soil and water pollution on food safety and health risks in China. *Environment International*.

[41] Mahvi A. H., Karyab H. (2007). Risk assessment for microbial pollution in drinking water in small community and relation to diarrhoea disease. *American-Eurasian Journal of Agricultural and Environmental Science*.

[42] Marathe N. P., Pal C., Gaikwad S. S., Jonsson V., Kristiansson E., Larsson D. J. (2017). Untreated urban waste contaminates Indian river sediments with resistance genes to last resort antibiotics. *Water Research*.

[43] Martineau F., Picard F. J., Lansac N. (2000). Correlation between the resistance genotype determined by multiplex PCR assays and the antibiotic susceptibility patterns of Staphylococcus aureus and Staphylococcus epidermidis. *Antimicrobial Agents and Chemotherapy*.

[44] McLellan S. L., Eren A. M. (2014). Discovering new indicators of fecal pollution. *Trends in Microbiology*.

[45] McLellan S. L., Daniels A. D., Salmore A. K. (2001). Clonal populations of thermotolerant Enterobacteriaceae in recreational water and their potential interference with fecal Escherichia coli counts. *Applied and Environmental Microbiology*.

[46] Mezrioui N., Baleux B. (1994). Resistance patterns of E. coli strains isolated from domestic sewage before and after treatment in both aerobic lagoon and activated sludge. *Water Research*.

[47] Moges F., Endris M., Belyhun Y., Worku W. (2014). Isolation and characterization of multiple drug resistance bacterial pathogens from waste water in hospital and non-hospital environments, Northwest Ethiopia. *BMC Research Notes*.

[48] Newman M. J., Frimpong E., Donkor E. S., Opintan J. A., Asamoah-Adu A. (2011). Resistance to antimicrobial drugs in Ghana. *Infection and drug resistance*.

[49] Nkansah M. A., Boadi N. O., Badu M. (2010). Assessment of the quality of water from hand-dug wells in Ghana. *Environmental Health Insights*.

[50] Nogueira G., Nakamura C. V., Tognim M. C. B., Filho B. A. A., Filho B. P. D. (2003). Microbiological quality of drinking water of urban and rural communities, Brazil. *Rev Saúde Pública*.

[51] Obiri-Danso C. A., Weobong C. A., Jones K. (2005). Aspects of health-related microbiology of the Subin, an urban river in Kumasi, Ghana. *Journal of Water and Health*.

[52] Odonkor S. T., Ampofo J. K. (2013). Escherichia coli as an indicator of bacteriological quality of water: an overview. *Microbiology Research*.

[53] Odonkor S. T., Mahami T. (2020). _Escherichia coli_ as a Tool for Disease Risk Assessment of Drinking Water Sources. *International Journal of Microbiology*.

[54] Odonkor S. T., Addo K. K. (2018). Prevalence of multidrug-resistant Escherichia coli isolated from drinking water sources. *International journal of microbiology*.

[55] Omari S., Yeboah-Manu D. (2012). The study of bacterial contamination of drinking water sources: a case study of Mpraeso, Ghana. *The Internet Journal of Microbiology*.

[56] Opintan J. A., Newman M. J. (2017). Prevalence of antimicrobial resistant pathogens from blood cultures: results from a laboratory based nationwide surveillance in Ghana. *Antimicrobial Resistance & Infection Control*.

[57] Osunla C., Okoh A. (2017). Vibrio pathogens: a public health concern in rural water resources in sub-Saharan Africa. *International Journal of Environmental Research and Public Health*.

[58] Owusu P. A., Asumadu-Sarkodie S., Ameyo P. (2016). A review of Ghana’s water resource management and the future prospect. *Cogent Engineering*.

[59] Pan M., Chu L. M. (2018). Occurrence of antibiotics and antibiotic resistance genes in soils from wastewater irrigation areas in the Pearl River Delta region, southern China. *Science of the Total Environment*.

[60] Parveen S., Murphee R. L., Edmiton L., Kaspar C. W., Portier K. M., Tamplin M. L. (1997). Association of multiple-antibiotic resistance profiles with point and nonpoint sources of Escherichia coli in Apalachicola Bay. *Applied and Environmental Microbiology*.

[61] Petit F., Clermont O., Delannoy S. (2017). Change in the structure of Escherichia coli population and the pattern of virulence genes along a rural aquatic continuum. *Frontiers in Microbiology*.

[62] Podschun R., Ullmann U. (1998). Klebsiella spp. as nosocomial pathogens: epidemiology, taxonomy, typing methods, and pathogenicity factors. *Clinical Microbiology Reviews*.

[63] Prabhu D., Pandian R. S., Vasan P. T. (2007). *Pathogenicity, antibiotic susceptibility and genetic similarity of environmental and clinical isolates of Vibrio cholerae*.

[64] Qiao M., Ying G. G., Singer A. C., Zhu Y. G. (2018). Review of antibiotic resistance in China and its environment. *Environment International*.

[65] Quiroz K. L., Rodriguez N. G., Murinda S., Ibekwe M. (2018). *Determination of the Water Quality of a Constructed Wetland Monitoring Fecal Indicator Bacteria*.

[66] Resende A. C. B., de Bastos Ascenso Soares R., Santos D. B., Montalvão E. R., do Carmo Filho J. R. (2009). Detection of antimicrobial-resistant Gram-negative bacteria in hospital effluents and in the sewage treatment station of Goiânia Brazil. *O Mundo da Saúde*.

[67] Rodrigues C., Cunha M. Â. (2017). Assessment of the microbiological quality of recreational waters: indicators and methods. *Euro-Mediterranean Journal for Environmental Integration*.

[68] Schafhauser B. H., Kristofco L. A., de Oliveira C. M. R., Brooks B. W. (2018). Global review and analysis of erythromycin in the environment: occurrence, bioaccumulation and antibiotic resistance hazards. *Environmental Pollution*.

[69] Shahina J., Sandhiya D., Rafiq S. (2020). Bacteriological quality assessment of groundwater and surface water in Chennai. *Nature Environment & Pollution Technology*.

[70] Tambekar D. H., Dhanorkar D. V., Gulhane S. R., Khandelwal V. K., Dudhane M. N. (2006). Antibacterial susceptibility of some urinary tract pathogens to commonly used antibiotics. *African Journal of Biotechnology*.

[71] Team R. C. (2018). *R: A Language and Environment for Statistical Computing*.

[72] Wangai F. K., Masika M. M., Lule G. N. (2019). Bridging antimicrobial resistance knowledge gaps: the East African perspective on a global problem. *PLoS One*.

[73] World Health Organization (1997). *Guidelines for Drinking-Water Quality: Volume 2: Surveillance and Control of Community Supplies*.

[74] Who (2004). *Guidelines for Drinking Water Quality: Recommendations*.

[75] Who (2006). *Guidelines for Drinking- Water Quality: Incorporating First Addendum*.

[76] Wikler M. A. (2006). Methods for dilution antimicrobial susceptibility tests for bacteria that grow aerobically: approved standard. *CLSI (NCCLS)*.

[77] Xu L., Ouyang W., Qian Y., Su C., Su J., Chen H. (2016). High-throughput profiling of antibiotic resistance genes in drinking water treatment plants and distribution systems. *Environmental Pollution*.

[78] Xue X., Cashman S., Gaglione A. (2019). Holistic analysis of urban water systems in the Greater Cincinnati region:(1) life cycle assessment and cost implications. *Water research X*.

[79] Yevutsey S. K., Buabeng K. O., Aikins M. (2017). Situational analysis of antibiotic use and resistance in Ghana: policy and regulation. *BMC Public Health*.

[80] Zhang C., Qiu S., Wang Y. (2013). Higher isolation of NDM-1 producing Acinetobacter baumannii from the sewage of the hospitals in Beijing. *PLoS One*.

